The article "Effects of Running Surface Stiffness on Three-Segment Foot Kinematics Responses with Different Shod Conditions" was published in 2021. Journal: Appl Bionics Biomech.

# Effects of Running Surface Stiffness on Three-Segment Foot Kinematics Responses with Different Shod Conditions

**DOI:** 10.1155/2021/8842591

**Published:** 2021-01-30

**Authors:** Noor Arifah Azwani Abdul Yamin, Khairul Salleh Basaruddin, Ahmad Faizal Salleh, Mohammad Shahril Salim, Wan Zuki Azman Wan Muhamad

**Affiliations:** ^1^School of Mechatronic Engineering, Universiti Malaysia Perlis, 02600 Pauh Putra, Perlis, Malaysia; ^2^Medical Device and Life Sciences Cluster, Sports Engineering Research Center (SERC), Universiti Malaysia Perlis, 02600 Pauh Putra, Perlis, Malaysia; ^3^Institute of Engineering Mathematics, Universiti Malaysia Perlis, 02600 Pauh Putra, Perlis, Malaysia

## Abstract

**Objective:**

The aim of this study was to investigate the effects of surface stiffness on multisegment foot kinematics and temporal parameters during running.

**Methods:**

Eighteen male subjects ran on three different surfaces (i.e., concrete, artificial grass, and rubber) in both heeled running shoes (HS) and minimal running shoes (MS). Both these shoes had dissimilar sole profiles. The heeled shoes had a higher sole at the heel, a thick base, and arch support, whereas the minimal shoes had a flat base sole. Indeed, the studied biomechanical parameters responded differently in the different footwear during running. Subjects ran in recreational mode speed while 3D foot kinematics (i.e., joint rotation and peak medial longitudinal arch (MLA) angle) were determined using a motion capture system (Qualysis, Gothenburg, Sweden). Information on stance time and plantar fascia strain (PFS) was also collected.

**Results:**

Running on different surface stiffness was found to significantly affect the peak MLA angles and stance times for both HS and MS conditions. However, the results showed that the joint rotation angles were not sensitive to surface stiffness. Also, PFS showed no relationship with surface stiffness, as the results were varied as the surface stiffness was changed.

**Conclusion:**

The surface stiffness significantly contributed towards the effects of peak MLA angle and stance time. These findings may enhance the understanding of biomechanical responses on various running surfaces stiffness in different shoe conditions.

## 1. Introduction

Running is a popular activity that has been connected to various clinical benefits [1]. However, based on analyses of etiology, running is also associated with increased risk of major chronic injuries among runners [2]. Any misalignment of the foot segment during running especially in the stance phase may contribute to foot and ankle injury, which is implicated in the etiology of the injury [3]. Foot misalignment that causes joint twisting can lead to inflammation of the ligament, such as plantar fascia. Plantar fascia inflammation contributes to plantar fasciitis, which is a known common injury for runners. Foot injuries that have occurred can be evaluated by kinematic or kinetic measurement. The progression of several pathologies, such as tibial stress syndrome or Achilles tendonitis, has been related to excessive coronal and/or transverse plane motion of the foot, which were identified using kinematic measurement [4].

Several studies have reported the effects of running surface on lower extremity kinematic parameters during running [5–12]. It was noted that surface effect has been investigated in terms of different running surface properties, including irregularity, inclination, and stiffness. In a previous surface stiffness investigation, Stergiou and Bates [12] studied the effects of surface hardness on the relationship between subtalar and knee joint function in an investigation that involved knee and ankle measurements. It was reported that there is a strong inner relationship between pronation and tibial rotation of knee joint function. The result also showed that there is a significant difference in the impact force, but no significant difference for kinematic and temporal parameters for each joint. Dixon et al. [11] evaluated the biomechanical response of the runner's heel striking the surface-to-surface hardness changes in a study that involved mechanics measurements of the hips, knees, and ankles. The results found that the kinematic responses of group analysis showed no significant differences, but varied in the responses of joint angle, peak joint angle, and peak joint angular velocities of the hip, and knee and ankle to surface stiffness for individual analysis. Similarly, Hardin et al. [10] investigated the kinematic adaptations of the hips, knees, and ankles influenced by surface stiffness during running. It was found that the knee flexion and the maximal hip flexion decreased with respect to the increasing surface stiffness, but the peak angular velocities of all investigated joints increased. Generally, there is a notable paucity of studies describing how the surface affects foot kinematics, especially during running.

In addition, although these prior studies have been focused on lower extremity kinematics that are affected by running surface, foot mechanics as a three-segment factor has not been established. In fact, most of these studies investigated the foot as a single, rigid segment. Three-segment foot mechanics were utilized by Sinclair et al. [13] in evaluating the effects of surface inclination on foot kinematics. The study was done by effectively overcoming the limitations of viewing the foot as a single rigid segment. It was reported that the rearfoot performed significantly greater plantar flexion on the varied incline conditions although the multisegment foot kinematics waveform measured as a function were quantitatively similar. The multisegment analysis was shown to be capable of prevailing over a single rigid segment or vector assumption of a foot at standard gait analysis and may better allow researchers to consider deformity in dynamic modelling. The relation of each appointed foot segment was also accurately evaluated with multisegment analysis during motion. Furthermore, constructive awareness of segmental foot kinematics was also offered when using multisegment analysis.

Furthermore, as suggested by Fu et al. [14], hard surfaces result in higher injury risks as compared to soft surfaces. Therefore, surface stiffness was included as a principal property to be taken into account during the selection of running surfaces. The biomechanical response of running was modified according to surface stiffness that may generate high impact force by adjusting and compensating the lower extremity. In order to maintain the impact force during running, the landing pattern was altered unconsciously to be slightly softer when running on hard surfaces and vice versa. These alterations are also known as kinematic adjustment. However, kinematic adjustment may also contribute to injuries, such as ankle and foot sprains. Risk factors for injuries related to kinematic adjustment were not discussed in detail as insufficient information was provided. Although some studies have been conducted to examine the effect of running conditions (i.e., running surface and shod condition) on kinematic and kinetic responses, these studies were limited to a single rigid segment foot model. However, the single rigid segment foot model may not produce adequate information as it is limited to a single segment of the foot. The application of dynamic modelling in terms of multisegments is probably needed. This is in order to investigate the relationship of foot segments in kinematic adaptation during running in detail. Therefore, further research on kinematic adaptation using multisegment modelling is required to enhance knowledge on injury risk during running on different surfaces.

To date, there has been no experimental evidence on the effects of surface stiffness on multisegment foot mechanics. In addition, prior studies have demonstrated that the adjustment of running mechanics is influenced by the type of running shoes or footwear [15, 16]. Therefore, the purpose of the current study is to investigate the effects of surface stiffness on multisegment kinematics of the foot during running with two different types of footwear.

## 2. Methodology

### 2.1. Participants

Eighteen healthy male individuals from a university population were recruited for this study and had a mean age of 24 ± 1.2 years old, height of 172 ± 2.7 cm, and body mass of 67 ± 6.7 kg. All the participants fell within the normal body mass index (BMI) category. In order to avoid any dissimilarity in the movement and amount of effort required to conduct assigned tasks, individuals with prior musculoskeletal injuries or orthopedic abnormalities have been removed from the analysis. The Ethics Committee under University Malaysia Perlis approved this study, and each participant was required to fill out a provided survey and sign a consent form prior to the experiment.

### 2.2. Equipment and Devices

Five Oqus motion capture cameras (Qualysis, Gothenburg, Sweden) set at a frequency of 200 Hz and two force plates (Bertec Corp., Columbus, Ohio, USA) were used in the experiment. The equipment arrangement is shown in Figure 1.

Markers with diameters of 20 mm and 15 mm covered with reflective tape were used. Twelve reflective markers were attached on anatomical landmarks in accordance with Leardini et al. [17] foot model protocols to assign the anatomical segment frames of the calcaneus, midfoot, and metatarsus. Markers were placed at the base of the first metatarsal (FMB), the head of the first metatarsal (FMH), the base of the second metatarsal (SMB), the head of the second metatarsal (SMH), the base of the fifth metatarsal (VMB), and the head of the fifth metatarsal (VMH) for metatarsus segment. In the midfoot segment, the landmark of markers was placed at the most medial apex of the tuberosity of the navicular (TN), while for the calcaneus segment, the upper central ridge of the calcaneus posterior surface (CA), the lateral apex of the peroneal tubercle (PT), the most medial apex of the sustentaculum tali (ST), and the medial malleolus (MANK) and lateral malleolus (LANK) were involved. Markers were digitized using a Qualysis motion capture system (Qualysis, Gothenburg, Sweden) and exported to a visual three-dimensional (3D) software (C-motion, Germantown, USA). Each participant wore two types of running shoes: minimal shoes (MS) and heeled shoes (HS) throughout the experiment. Both of these shoes have a dissimilar sole profile. The heeled shoe has a higher sole at the heel (heel drop), whereas the minimal shoe has a flat sole. It has been reported that the biomechanical parameters responded differently to the type of shoes during running [18].  Figure 2 shows the profile of running shoes that were used in the experiment.

The part of the shoes which overlapped with the region for marker placement was removed to ensure the markers were directly attached to the skin. The attachment of the markers is as presented in Figure 3.

Runway surfaces were selected based on common surfaces used for recreational running with different degrees of stiffness, which were concrete, rubber, and artificial grass. Stiffness tests on all surfaces were conducted according to the American Society for Testing Materials (ASTM) standard ASTM F2117-10 [19]. In this test, a basketball was dropped from a height of 2 m, and the vertical rebound height of the ball was recorded for each surface. Based on this simple experiment, the concrete surface was found to be the stiffest surface, with a vertical rebound of 103.04 ± 3.5 cm, while the artificial grass surface was found to be stiffer than the rubber surface with vertical rebounds of 97.80 ± 2.9 cm and 79.97 ± 4.4 cm, respectively. All selected running surfaces were placed on a similar wooden platform in the laboratory. The schematic diagram is shown in Figure 4.

### 2.3. Procedure

Prior to the experiment, the participants were instructed to run on the track to familiarise themselves with the conditions of the experiment. When the participants stood upright in a double-leg support pose, a static condition reference was recorded in order to identify the neutral location of the joint in each person [17]. Once the static position measurements were recorded, each participant was asked to run at their comfortable speed to reflect recreational running on the three different runway surfaces (i.e., concrete, artificial grass, and rubber) with dimensions of 7 m length and 1 m width. The measurements taken were approved to be recorded if all the markers were clearly captured and the right foot contacted with the force plate without any apparent alteration in the running stride. The participants were first asked to run wearing HS, and then, the procedure was repeated with MS.

### 2.4. Data Analysis

In order to remove the effect of other variables besides surface hardness, a screening process on the foot strike pattern of each participant was performed [20]. The foot strike pattern was identified mainly based on the angle of incidence (AOI), which is the angle between the horizontal plane and the line formed by the fifth metatarsal head and lateral malleolus. The foot strike pattern was evaluated in accordance with the calculation provided by Miller et al. [21]. An AOI of 0° indicated midfoot strike (MFS), whereas an AOI of more than 0° indicated a forefoot strike (FFS), and an AOI of less than 0° indicated a rearfoot strike (RFS), when normalized to the AOI measured during the standing posture, respectively. In order to ensure data accuracy, the foot strike pattern was further checked using visual analysis with the Qualysis software. However, in order to exclude potentially influencing factors other than the surface hardness, only the heel strike pattern performed by each participant was evaluated in the experiment.

During analysis, the trajectories of the reflective markers were filtered at 12 Hz using a low-pass filter [22]. Stance phase angles were computed using an XYZ cardan sequence for a motion of the midfoot with respect to the calcaneus (i.e., calcaneus-midfoot), the metatarsus with respect to midfoot (i.e., midfoot-metatarsal), and also the metatarsus with respect to the not-adjacent calcaneus (i.e., calcaneus-metatarsal). Euler angles were utilized to evaluate 3D rotations of the foot segments relative to each other. The parameters measured and analyzed were as follows: (1) range of motion (ROM) or the angle of rotation of each foot segment during overall stance phase and midstance phase, (2) stance time or the duration of time needed for participants to complete one cycle of stance phase, (3) plantar fascia strain or the change in length during the stance phase divided by the original length of the relative position distance between the calcaneus and first metatarsal markers, and (4) medial longitudinal arch (MLA) or the angle subtended by the combination of a line from the marker on the FMH to the TN and another line from the ST to the TN marker.

Means and standard deviations of the parameters measured were determined for each surface hardness condition. The means and standard deviations were evaluated in a normality test using the Shapiro-Wilk test, which showed that the obtained data was not normally distributed. Differences for each parameter measured were evaluated using the nonparametric test; the two-way Kruskal-Wallis test with statistical significance was accepted at *p* < 0.1. The Kruskal-Wallis test was selected as it is the most suitable test in statistical analysis for investigating the differences of two or more means for abnormally distributed data. Statistical Package for Social Science (SPSS) version 17.0 (IBM, Armonk, NY, USA) was utilized to perform the statistical analysis.

## 3. Results

### 3.1. Joint Rotation of Three-Foot Segments

Figure 5 shows the joint rotation angle in the stance phase during HS running. The 3D rotation patterns of joint segments of HS running for the calcaneus-metatarsal and midfoot-metatarsal joint segments were found to be similar for the frontal, transverse, and sagittal planes on all surfaces. Both joint segments performed inversion, adduction, and plantar flexion, as presented in Figures 5(a), 5(b), 5(c), 5(g), 5(h), and 5(i), respectively. In addition to these findings, artificial grass was also shown to be the highest in both frontal and sagittal planes for midfoot-metatarsal joint segments as illustrated in Figures 5(g) and 5(i), respectively. While for the calcaneus-midfoot joint segment during HS running, the inversion was performed in the frontal plane as shown in Figure 5(d), while dorsiflexion was demonstrated in the sagittal plane on all surfaces as presented in Figure 5(f). However, as can been seen in Figure 5(e), the calcaneus-midfoot joint segment is slightly adducted where the angle of rotation is almost zero during running on artificial grass, but there is slight abduction in the transverse plane during running on rubber and concrete surfaces. Although the results showed different values on the joint angles for each plane, the overall waveforms of kinematic measurement were still of similar patterns as seen in the figures. As such, surface hardness seemed to not affect HS running (*p* < 0.05).

Furthermore, MS running was found to be in a uniform trend, and the surface hardness was found to not affect the joint rotations. A clear trend for each plane for all joint segments of MS running can be seen in Figure 6. Inversion was performed in the frontal plane (Figures 6(a), 6(d), and 6(g)), and adduction was completed in the transverse plane (Figures 6(b) and 6(e)), except for the midfoot-metatarsal joint segments in which the use of the concrete surface contributed to a slight adduction as seen in Figure 6(h). Note that the rubber surface had the lowest inversion compared to the other two surfaces for the midfoot-metatarsal joint segment. Also, interestingly, plantar flexion was demonstrated in the case of the calcaneus-metatarsal and midfoot-metatarsal joint segments as presented in Figures 6(c) and 6(i), respectively. As can be seen in Figure 6(f), dorsiflexion was performed for the calcaneus-midfoot joint segment on all running surfaces.

Together, these results provide important insight into joint rotation at the midstance phase, which was statistically analyzed using the Kruskal-Wallis (one-way) method. The joint rotations during midstance of HS and MS running showed no significant difference in the motion of the segments due to surface hardness. The results of the statistical analysis are shown in Table 1 for HS running and Table 2 for MS running. The results showed that all kinematic variables obtained in the study were not statistically significant with *p* > 0.1.

Peak medial longitudinal arc (MLA) angle and MLA angle were relative to a range of motion (ROM). The results of peak medial longitudinal arch (MLA) angle on all running surfaces in both shod conditions are presented in Table 3. Interestingly, for HS running conditions, the highest value of peak MLA angle was achieved during running on the concrete surface, which was followed by artificial grass and rubber surfaces, with both showing similar results. However, the highest value of peak MLA for MS running conditions was achieved on artificial grass, followed by on concrete and lastly on rubber. From the information displayed in Table 3, it can be observed that the peak MLA angle of each running condition was not affected by the increase of surface hardness. It is also shown that there was a significant difference in HS running with *p* = 0.057 (*p* < 0.1), while there was no significant difference in MS running condition. Furthermore, in relation to the range of motion (ROM) in which the angular displacement from foot strike to peak angle was measured, there was also no relationship of MLA with the surface hardness observed for each running condition, as shown in Table 3. The MLA relative to the ROM was the highest during running activity on the concrete surface in both shod conditions, while the MLA relative to ROM was the lowest during running on artificial grass during MS running with a value of 4.623 ± 3.128. On the other hand, the MLA relative to ROM was the lowest during running on rubber in HS with a value of 5.358 ± 2.58 (*p* = 0.109).

### 3.2. Plantar Fascia Strain

With respect to Table 3, the analysis of the obtained data using the Kruskal-Wallis test showed no statistically significant difference of plantar fascia strain between each running surface with *p* = 0.977 (*p* > 0.1) for MS and *p* = 0.949 (*p* > 0.1) for HS. The plantar fascia strain was lowest when running on rubber at 89.434 ± 17.5 × 10^−3^ under MS conditions and lowest when running on concrete at 70.632 ± 21.2 × 10^−3^ under HS conditions. However, both shod conditions recorded the highest plantar fascia strain during running on the artificial grass surface, with values of 91.195 ± 22.8 × 10^−3^ and 78.630 ± 35.1 × 10^−3^ under MS and HS conditions, respectively.

### 3.3. Temporal Parameter

Stance time was calculated at the instant of foot strike until toe off during running on each surface. Under MS condition, running on concrete had the lowest stance time, whereas running on rubber had the highest stance time. Therefore, it can be said that MS condition stance time is related to surface hardness. However, under HS condition, the lowest stance time was recorded when running on artificial grass, and the highest was recorded when running on concrete. Interestingly, it was found that there was a statistically significant difference for the comparison of stance times, which was significant at *p* = 0.092 and *p* = 0.090 (*p* > 0.1) for running under MS and HS conditions, respectively.

## 4. Discussion

The aim of the present study was to determine the effects of surface stiffness on foot segment kinematics, PFS, peak MLA, and temporal parameters during running with MS and HS. Surface stiffness was found to significantly affect the peak MLA angle during HS running, where the highest peak MLA angle was obtained on a concrete surface, followed by artificial grass and rubber surfaces (*p* > 0.1), whereas there was no significant difference in the peak MLA angle during MS running on all surfaces. The peak MLA angle response was shown to be consistent in trend regardless of shod conditions. However, there was no relationship between peak MLA angle and surface stiffness. In addition, the MLA angle relative to the ROM of the stance phase as well as foot segment joint rotation was also found to be not related to surface stiffness. The foot segment joint rotation was shown to be in an almost similar pattern of motion in each plane for both shod conditions during running on each surface. The findings of these kinematic parameters further support the results reported by previous studies, which investigated the kinematic of the foot as a single rigid body [10, 11]. Dixon et al. [11] reported that there was no statistical difference in kinematic variables when the peak of the angle was measured. In addition, these results also corroborate the findings of Hardin et al. [10], who found that kinematic adaptation on surfaces only occurs at the hip and knee, but not at the ankle. Adaptation to variations in surface hardness primarily involves the kinematic changes of the hip and knee joints instead of the ankle or the foot. Still, there may be a small involvement of the ankle and the foot in kinematic adjustment for the purpose of adapting to various surfaces. Kinematic adjustment of leg stiffness was conducted to accommodate surface stiffness [23].

Moreover, it was found that the highest value of plantar fascia strain (PFS) was achieved during running on artificial grass for both shod conditions. The recurring manner of MLA angle with respect to shod conditions can also be seen in the PFS parameters, even though the PFS did not demonstrate a regular pattern with respect to surface hardness. Both peak MLA angle and PFS had the highest and lowest values during MS and HS running conditions, respectively. The plantar fascia is associated with MLA through a “windlass mechanism” [24]. The “windlass” words which are described as a tightening rope or cable are simulated by plantar fascia that is connected to the calcaneus and metatarsophalangeal joint. Due to dorsiflexion, the distance between calcaneus and metatarsal is reduced by the winding of the plantar fascia during the propulsive phase in the movement of gait [24]. As such, the reduced length of the plantar fascia due to dorsiflexion movement is believed to be the fundamental quality of the windlass mechanism [25]. Therefore, the results obtained in the present study further explained the windlass mechanism; that is, when PFS is longer, the MLA angle is increased due to the demotion of MLA.

The foot kinematics position and orientation in the present study were investigated as three segments. This analysis, which utilized optical tracking equipment, can be considered to be an advanced method in dynamic modelling for the purpose of defining the movement of segments of body parts. Previously published studies investigating foot kinematics during running generally using either two-dimensional (2D) or 3D systems treated the foot as a single rigid body or as two segments, respectively [10, 11, 26–28]. Multisegment analysis is capable of prevailing over a single segment assumption of the foot by common gait analysis and assisting with a better demonstration of deformity in dynamic modelling, as well as providing more detailed information on the relationship of the movement of the foot segments during running [29].

The most striking finding was the fact that there was a relationship between stance time and surface hardness during running with MS instead of HS. During running with MS, it was shown that higher surface hardness resulted in lower stance time. In addition, there was a statistically significant difference in the stance time during running on the numerous surfaces for both shoe conditions. The relationship between stance time and surface hardness during running with MS agrees with the findings from some published studies [22, 30, 31] that found that stance time is longer when the runner is on a softer surface as compared with harder surfaces. Although these results are in agreement with some previous articles, the findings are inconsistent with those reported by Hardin et al. [10] and Hong et al. [32]. This disagreement can likely be explained by the use of different types of shoes, running velocity, and measurement method. In contrast to the earlier findings reported regarding the relationship of stance time and surface hardness, the disassociated relation when running with HS may be explained by the properties of the sole of the shoes (i.e., thickness and shape). The sole profile of HS leads to a greater ankle dorsiflexion angle compared to MS during running. A greater dorsiflexion of the ankle raises the knee flexion angle [33] which correlates to the running efficiency [34]. A higher flexion also could reduce the peak vertical ground reaction force [34] because the loadings at the knee and hip joints were decreased. As reported by Heiderscheit et al. [35], the reduction of these loadings is due to the increase of 5% to 10% of stride cadence. It was recorded that the higher stride cadence was associated with shorter stance time [36]. Therefore, a difference in the stance time can be observed in both types of footwear but less for the HS shoe.

Therefore, in general, it was found that the difference in terms of magnitude and the general trend of measured response parameter with respect to surface hardness and shod condition were not huge. A possible explanation for this might be due to the small differences in the levels of surface hardness determined according to the rebound height of the hardness test. Thus, the response of parameter measured in adaptation to the surface was found not to be sensitive to the small differences in surface hardness. However, although the differences were not obvious, there were some significant effects of surface hardness and shod conditions that were recognized from this study. The results obtained from this study are likely to be meaningful in terms of the aspect of the type of surface. This is because the difference of parameters investigated might be due to the different types of running surfaces rather than their hardness. Therefore, this study contributes a major role in determining surface and shod selection, in addition to the development of surfaces for various activities, including running.

A potential drawback of this study is that running movement was limited to recreational mode, which affected the range of surface hardness to only candidates that would be involved in this type of activity. In addition, this experiment was conducted with speed control ranging from 1.6 m/s to 2.4 m/s. The running speed was limited in accordance with the length of the indoor running track. The general findings of this study were all based on this speed range. Future work should include a greater variety of running activities, such as sprinting or long-distance running; hence, more surface types might provide additional evidence regarding the influence of running surfaces on biomechanical responses.

## 5. Conclusion

The present study provided additional insights on multisegment measurements of foot adaptation response during running with two different running shoes on different degrees of surface hardness. This study found that stance time was significantly affected by the different degrees of surface hardness for both shod conditions. However, generally, there was no relationship between surface hardness and kinematic parameters during running with both types of running shoes. Additionally, this study suggested that the variation in PFS was due to changes in the running surface for both shod conditions. Overall, the results of the present study suggested that surface hardness significantly affected peak the MLA angle and stance time. In short, these findings might enhance the understanding of biomechanical responses on various running surfaces in different shod conditions. This understanding should help in the selection of both running surface and shoes to improve performance and reduce injury risk. Performance improvement and injury risk during running are closely related to stance time, PFS, and peak MLA angle. Thus, from the results of this research, it is suggested to wear HS during running as it has the lowest stance time, PFS, and peak MLA angle. It is also suggested to run on an artificial grass surface in improving running performance but on a rubber surface in reducing the risk of injury.

## Figures and Tables

**Figure 1:** Layout of the experiment.

**Figure 2:** Profile of running shoes used in the experiment: (a) minimal shoe (MS), (b) heeled shoe (HS), and (c) sole profile of HS.

**Figure 3:** The marker placement: (a) marker placement, (b) marker attached during wearing cushion heeled running shoe, and (c) marker attached during wearing minimally.

**Figure 4:** Schematic diagram of running runaway.

**Figure 5:** Angle of joint rotation in the foot segment of heeled shoe (HS) running: (a) calcaneus-metatarsal (eversion/inversion), (b) calcaneus-metatarsal (abduction/adduction), (c) calcaneus-metatarsal (plantar/dorsi flexion), (d) calcaneus midfoot (eversion/inversion), (e) calcaneus-midfoot (abduction/adduction), (f) calcaneus-midfoot (plantar/dorsi flexion), (g) midfoot-metatarsal (eversion/inversion), (h) midfoot-metatarsal (abduction/adduction), and (i) midfoot-metatarsal (plantar/dorsi flexion).

**Figure 6:** Angle of joint rotation in the foot segment of minimal shoe (MS) running: (a) calcaneus-metatarsal (eversion/inversion), (b) calcaneus-metatarsal (abduction/adduction), (c) calcaneus-metatarsal (plantar/dorsi flexion), (d) calcaneus midfoot (eversion/inversion), (e) calcaneus-midfoot (abduction/adduction), (f) calcaneus-midfoot (plantar/dorsi flexion), (g) midfoot-metatarsal (eversion/inversion), (h) midfoot-metatarsal (abduction/adduction), and (i) midfoot-metatarsal (plantar/dorsi flexion).

**Table 1:** Joint rotation during midstance of HS running.

Angle of rotation		Rubber		Artificial grass		Concrete		*p* value
		Mean	SD	Mean	SD	Mean	SD	
Calcaneus-metatarsal	Eversion/inversion (°)	-14.741	3.14	-8.659	11.70	-15.20	6.92	0.532
	Abduction/adduction (°)	-18.793	6.49	-16.794	15.78	-20.173	6.74	0.738
	Dorsiflexion/plantarflexion (°)	-45.130	3.71	-48.692	6.83	-48.711	20.02	0.470

Calcaneus-midfoot	Eversion/inversion (°)	-14.038	4.98	-15.349	3.25	-10.431	5.24	0.130
	Abduction/adduction (°)	4.170	5.94	0.002	6.55	3.140	2.11	0.587
	Dorsiflexion/plantarflexion (°)	46.417	5.16	43.733	2.27	44.347	2.62	0.810

Midfoot-metatarsal	Eversion/inversion (°)	-10.656	5.39	-13.413	3.03	-11.548	6.76	0.581
	Abduction/adduction (°)	-6.790	6.08	-5.150	6.40	-9.669	8.44	0.751
	Dorsiflexion/plantarflexion (°)	-81.298	17.60	-88.783	7.62	-83.155	6.90	0.524

**Table 2:** Joint rotation during midstance of MS running.

Angle of rotation		Rubber		Artificial grass		Concrete		*p* value
		Mean	SD	Mean	SD	Mean	SD	
Calcaneus-metatarsal	Eversion/inversion (°)	-13.622	1.96	-15.567	3.02	-15.967	5.48	0.421
	Abduction/adduction (°)	-20.096	6.74	-16.423	6.95	-15.348	5.64	0.347
	Dorsiflexion/plantarflexion (°)	-52.956	6.97	-55.081	5.11	-51.536	10.23	0.751

Calcaneus-mid foot	Eversion/inversion (°)	-15.457	2.57	-14.366	2.60	-15.324	2.76	0.884
	Abduction/adduction (°)	-1.562	4.77	-1.898	6.14	-1.461	4.50	0.949
	Dorsiflexion/plantarflexion (°)	31.650	6.09	32.416	3.42	31.138	3.90	0.849

Midfoot-metatarsal	Eversion/inversion (°)	-13.622	1.96	-15.567	3.02	-15.967	5.48	0.421
	Abduction/adduction (°)	-20.096	6.74	-16.423	6.95	-15.348	5.64	0.347
	Dorsiflexion/plantarflexion (°)	-52.956	6.97	-55.081	5.11	-51.536	10.23	0.751

**Table 3:** Effects of running surface on peak MLA, MLA, relative to ROM, PFS, and stance time.

		Rubber		Artificial grass		Concrete		*p* value
		Mean	SD	Mean	SD	Mean	SD	
MS	Peak MLA angle (°)	166.242	3.319	167.745	3.046	167.518	6.366	0.630
	MLA relative ROM (°)	7.648	3.411	4.623	3.128	8.290	2.045	0.109
	Plantar fascia strain (×10^−3^)	89.434	32.54	91.195	22.80	89.854	21.17	0.977
	Stance time (×10-^3^ s)	278.3	25.2	254.2	12.4	250.0	22.4	0.092^∗^

HS	Peak MLA angle (°)	156.743	3.12	157.175	3.57	161.318	4.02	0.057^∗^
	MLA relative ROM (°)	5.358	2.58	5.998	3.10	7.135	1.56	0.414
	Plantar fascia strain (×10^−3^)	71.255	17.50	78.630	35.03	70.632	17.83	0.949
	Stance time (×10^−3^ s)	260.8	9.2	247.5	24.0	278.3	34.9	0.090^∗^

## Data Availability

Readers can request the corresponding author for motion capture datasets.
